RETRACTED

# Reflections on the Discipline Construction Environment of World Literature and Comparative Literature in the Era of Big Data Analysis

**DOI:** 10.1155/2022/2786610

**Published:** 2022-09-07

**Authors:** Wen Xu

**Affiliations:** School of Chinese Language and Literature, Suzhou University of Science and Technology, Suzhou 215000, China

## Abstract

Comparative literature and world literature were originally two independent disciplines, but now they are merged into one. In the era of big data, building an efficient information management method is one of the important contents of university reform. Based on the construction of comparative literature and world literature, this paper applies the DSS (Decision Support System) structure based on data warehouse to the construction of comparative literature and world literature, and constructs the DSS structure of comparative literature and world literature. The related knowledge of DM (data mining) is used for research, and the application design and implementation process of DM are introduced into the subject quality evaluation system. The research shows that the experimental results of NB (Naive Bayes) algorithm will not take too long, about 56.08 s, and the compression ratio is 0.897, when the parameters are basically the same. This model can effectively help schools to analyze data and make decisions, and improve the level of information construction in schools.

## 1. Introduction

Comparative literature, foreign literature, and world literature—as well as each of their unique characteristics, research areas, and relationships—have long been hotly debated subjects in China's academic and educational communities. The combination of comparative literature and world literature creates “comparative literature and world literature,” which not only expands on comparative literature's research ideas but also gives it a theoretical foundation and a large stage on which to grow. The majority of colleges and universities still divide comparative and foreign literature instruction into two parts for independent study, which, in part, undermines the discipline's systematic nature and divides the requirements for the integration of China and the West. This is a significant development in both comparative and world literature. Of course, there are ferocious debates within this field of study, but progress has always been made in that direction.

Every science needs to have a clear place in the scientific encyclopedia. It is difficult to come to a consensus on what comparative literature is among the literary studies disciplines because it is so debatable. We can quickly locate this feature by looking back at the development of comparative literature [1, 2]. Some academics believe that this definition of “contemporary literature” is illogical because it conflicts with recent studies on the subject. Others believe it still has value as the term “expedient measure” [3]. The evolution of translation is integral to the history of foreign literature compilation. Notably, the majority of Chinese translations of foreign literary works from the first half of the 20th century have a strong utilitarian tone indicative of enlightenment. According to some studies, comparative literature iconography primarily examines the nation's “other image” and “self-image,” that is, the nation as it appears in literary creations, literary history, and literary criticism [4]. The goal of image research is to understand how images are created, how they change over time, and how they are influenced. The nation's limitations and one-sidedness are becoming more and more impractical, so numerous national and local literatures have combined to create a type of world literature [5]. The global exchange of cultures has, on the other hand, been greatly facilitated by the growth of modern media, particularly the Internet's invention and widespread use, and at the same time, the public now has access to a variety of information sources and cultural options.

RETRACTED

If comparative literature and world literature merge into an integrated disciplineand if this operation is reasonable, it will be the focus of researchers in related fields. At the same time, the research and compilation of world literature also has the ideology of comparative literature. Only by making full use of the method of comparative literature can we accurately and scientifically evaluate the literary content of each nation, and then determine its status. In the world literature, we promote the excellent literary content to spread all over the world forever. In the era of big data, DM (data mining) technology [6], as a new multidisciplinary subject, is increasingly applied to research fields, especially in the field of information analysis [7]. Systematic study and study of world literature can help us understand the world, and promote our communication and integration with people all over the world; At the same time, because we take the whole world literature as the frame of reference, our value, significance, and characteristics of Chinese literature will be reduced, and our understanding of Chinese literature will be clearer and deeper. Therefore, based on the key disciplines and degree management information systems and their data in colleges and universities, a networked computer system with comprehensive analysis and decision-making ability should be established to adapt to the new thinking of comparative literature and world literature discipline construction decision-making.

RETRACTED

Research innovation: (1) By introducing the communication theory, this paper opens up a new horizon for the study of comparative literature images, and helps to enrich the research methods and perspectives of image studies, broaden the research fields of image studies, and make the scale and depth of image studies develop in depth. (2) Based on the background of comparative literature and the construction of world literature discipline, this paper puts forward a DSS solution based on the data warehouse in the developed information system, and analyzes the tacit knowledge in comparative literature and the data in the construction system by using DM technology. Mining rules to provide decision-making opinions for decision-makers in colleges and universities has certain practical reference significance.

## 2. Related Work

### 2.1. Related Research on Discipline Construction

The fact that literature precedes world literature does not mean that comparative literature can replace world literature. Literature is “world” literature, not just “comparative” literature. Literature in the world has its own unique field and research scope. World literature refers to the literature of other countries except Chinese literature, including Europe, America, Asia, and Africa. The establishment of a discipline also outlines a unique field and scope for the discipline. Once this work is completed, it means that the discipline is becoming rigid and decadent, so it is necessary to break through the limitations and scope of the discipline.

Discipline establishment is the basis for the emergence and development of discipline-related research. The establishment of disciplines is accomplished through the deepening of academic research and the improvement of relevant educational systems. Discipline establishment is an institutional behavior that is closely related to the educational system. Briceo said, “When we re-examine the term comparative literature, we will find that it is a history of intense debate, which has lasted from the beginning of the century when the term appeared until today [8]. At the end of the century, the problems considered by the discipline theory of comparative literature “are still the same as those raised more than a century ago”, and they are still the fundamental problems and the “old” problems [9]. Larsen deepened his understanding of literature in general, while the unique perspective and methodology of comparative literature refreshed the traditional thinking of literary research, and also provided a new reference for other humanities and social disciplines [10].

RETRACTED

Zunshine found that humanistic spirit is the key to Chinese education [11]. Literature is an open and inclusive subject. The tolerant spirit and inclusive mentality of literature coincide with the concept of the new curriculum standard. Song's introduction of the concept of comparative literature into teaching can help us re-recognize ourselves in a diversified context, provide us with a vision of the other to examine ourselves, and inspire us to use a grand vision of world literature when reading and analyzing works [12]. In real work, how to embody the unique charm of foreign literary works and how to explore the humanity of foreign literary works, the quality of teachers themselves is even more important. Shaytanov pointed out the necessity, urgency, and feasibility of developing curriculum resources from the perspective of comparative literature [13]. The trend of comparative literature towards middle school is in line with the needs of the times.

### 2.2. Development and Present Situation of DSS Research

DSS (Decision Support System) is widely valued by scholars in various fields such as management science, data science, mathematics, and operational research. Among them, the human-computer interaction component is the interface between DSS and users. The user interaction component controls the operation of DSS, and the system also shows the decision support results to users through the interaction system. Components are used to build, store, and manage models, and also provide model operation language.

Wang put forward the three-component structure of DSS (dialogue component, data component, and model component), defined the basic components of DSS, and greatly promoted the development of DSS [14]. Hassan et al., through a problem in the application field of biological science, put forward a problem-solving method to obtain the chemical properties of compounds by mining the largest shared substructure in the structure set of compounds [15]. Kostuk and Willoughby through a problem in the application field of biological science put forward a problem-solving method to obtain the chemical properties of compounds by mining the largest shared substructure in the structure set of compounds [16]. In this algorithm, the input graph is compressed by the principle of minimum description length, and the column search based on greedy strategy is used as the search method, which can mine a very typical subgraph structure.

Kheterpal et al. believe that grid is a group of emerging technologies built on the Internet, forming a high-performance computing environment that can be used by each other, cooperated with each other, and transparent to multiple users, so as to gather scattered computing power, form supercomputing capability, and provide more resources, functions, and interactivity for scientists and ordinary users [17]. Cartwright et al. put forward an open DSS based on grid environment according to the open grid service architecture of grid. The remarkable feature of grid is to provide global resource and service sharing and collaborative work for solving complex problems [18]. Sim et al. call the grid information service provided by the grid environment to complete the query request of the decision maker; the service agent accepts the decision task given by the decision maker, and decomposes the decision task into subtasks according to the inquired decision service information [19]. Brown et al. think that grid technology has brought many new features to DSS, which can greatly strengthen the decision support ability for decision makers, such as abundant resources and powerful resource management, excellent parallelism, good scalability, high intelligence, unified data exchange form, and resource positioning mode [20].

RETRACTED

## 3. Methodology

### 3.1. DSS Construction of Comparative Literature and World Literature Discipline Construction

Future development opportunities for comparative and world literature are vast, and literary scholars must be fearless in putting forth their own viewpoints. Despite being combined into one discipline, they currently have a loose overall structure, and their development is largely independent. It is a waste of resources to carry out repetitive construction or low-level construction in the development of disciplines in China because there is insufficient investment in colleges and universities. The quality of colleges and universities varies, though, and the development of many colleges and universities has been hampered by the construction backlog brought on by a lack of funding. The comparison of national literature in oriental literature is also neglected in the field of comparative literature, as is the comparison of oriental literature with other regional or national literature. It appears that developing professionals in comparative literature is the primary goal of graduate study in comparative and world literature. New courses are being created by some enthusiastic teachers, who have even proposed the “teaching unit” model.

The research and teaching of any world literature must be “comparative”, because any researcher and teacher must stand in their own position, use their own eyes, and accumulate according to their own likes and dislikes, knowledge and culture. The whole social culture has always been a system that affects image communication. It is not difficult to see that the characteristics of communicators are similar to those of images, which makes it possible for image communication. Image is one of the contents of information. Information contains images, and the connotation of images is contained in the connotation of information. Therefore, in the process of image dissemination, the image must run through the whole social system. These theories are also applicable to the study of images in comparative literature, and they also play a guiding role in the process of image communication. These communication theories provide a theoretical basis for the development of image communication.

RETRACTED

The purpose of substructure discovery is to find novel and typical substructures. Let *S* be a substructure (individual), DL(*S*) be its description length, that is, the sum of the number of nodes and edges of *S*, and DL(*G|S*) be the sum of the number of nodes and edges of the graph obtained by replacing the instance of *S* in *G* with nodes. The fitness value of the individual *S* is defined as:

(1) $$\begin{array}{c} \text{fitness}\left(S\right)=\frac{1}{\text{DL}\left(S\right)+\text{DL}\left(G|S\right)}. \end{array}$$

The larger the compression degree of the visible substructure *S* to the input graph *G*, the better the substructure.

When the number of instances of an individual is 1, it has no development potential, because from the definition of compression ratio:

(2) $$\begin{array}{c} \text{compression}\_\text{ratio}\left(S\right)=\frac{\text{DL}\left(S\right)+\text{DL}\left(G|S|\right)}{\text{DL}\left(G\right)}. \end{array}$$

It can be seen that it basically does not compress the input graph. At this time, (*G|S*) is the graph obtained by replacing the instance in *S* with a point. When the number of instances in *S* is 1, *S* basically does not compress *G*. Such substructures should be immediately removed from the population and the newly generated unilateral substructure should be the used structure instead.

With the development of discipline construction, the monitoring workload is increasing day by day. How to design a perfect tracking system is the premise and guarantee of scientific and accurate tracking. The traditional database system can efficiently realize the functions of data input, modification, query, etc., but it cannot find the relationship between the data and lacks the means to extract the hidden knowledge behind the data, resulting in insufficient data. In order to meet the different processing depth requirements of different applications in database, multi-granularity in data warehouse is essential. The data organization structure in the data warehouse is divided into four levels, namely, initial level of detail, current level of detail, micro-integration, and high integration.

RETRACTED

The DSS structure of comparative literature and world literature discipline construction designed in this subject is established on the basis of fully combining the characteristics of discipline management in colleges and universities, the applicability of DSS, and the friendliness of users. The DSS framework of the discipline construction of comparative literature and world literature finally designed is shown in Figure 1.

The main characteristic of this system architecture is that it expands on the conventional DSS architecture by integrating data storage systems, database systems, and application systems. The enterprise database holds the acquired knowledge. Users can directly access the available knowledge from the knowledge base when making decisions about decision-making problems, which enhances the system's real-time performance. Save these memories and information in your brain. The brain uses prior experience to make the quickest decision possible when faced with a problem that needs to be solved.

The tasks of DM can be divided into two categories: describing tasks and predicting tasks. Descriptive mining mainly describes various properties in the database; predictive mining mainly infers and predicts data. Let *S* be the sample set, and *n* be the number of samples in it. The sample set is divided into *c* different classes, and each class *C*_*i*_ contains *n*_*i*_ samples. Then the information entropy of *S* divided into *c* classes is:

(3) $$\begin{array}{c} I\left(S_{1},S_{2},\ldots ,S_{m}\right)=-\sum_{i=1}^{m}p_{i}{\text{log}}_{2}\left(p_{i}\right). \end{array}$$

Among them, *p*_*i*_ is the probability of the sample in the *i*-th class *C*_*i*_, because the information is encoded in binary, so the entropy measurement of the encoding length is carried out in binary digits, so take 2 as the base of the logarithm.

When the attribute *A* is selected, the entropy of *S*_*v*_ classification is *E*(*S*_*v*_), and the definition of expected entropy is the weighted sum of *S*_*v*_ entropy of each subset. Namely:

(4) $$\begin{array}{c} E\left(S,A\right)=\sum \frac{\left|S_{v}\right|}{S}*E\left(S_{v}\right), \end{array}$$

where *E*(*S*_*v*_) represents the information entropy after dividing the samples in *S*_*v*_.

### 3.2. Subject Evaluation Method Based on DM

The incorporation of comparative literature and world literature appears to have been done with “cutting jobs and disciplines” in mind, according to the national higher education authority. Although comparative literature and world literature once belonged to the top fields of “foreign languages and literature” in the subject catalogue, many schools are located in Chinese departments in middle schools and universities of colleges and universities, according to the current state of postgraduate education in colleges and universities in China. The reason for this is that academic staff who teach and conduct research in foreign literature frequently only speak one or two foreign languages but are well-versed in the literature of those two countries. In order to distinguish similarities and differences between Chinese and foreign literary works and to better understand authors and their works, literary phenomena, and their laws, comparative literature must first identify the distinctive features of both types of literature.

RETRACTED

Chinese traditional literature and foreign literature, ancient and modern, Chinese and foreign are all included in the category of literature that is known as “world literature.” Chinese literature is even based on Chinese traditional literature and is thus integrated into world literature. Only a few courses on comparative literature's basic concepts are offered at some colleges and universities, which is insufficient to fulfill the goal of a thorough examination of the subject matter. Academic circles must continue to focus on the types of courses that should be offered to students majoring in comparative literature. Our discussion will therefore center on how to effectively use comparative literature knowledge to direct the teaching of foreign literature. There will undoubtedly be a wealth of new information in the popular philosophy, aesthetics, psychology, literature, art, and cultural studies fields today. As a result, the formation and dissemination of the people of a country are given special attention in the literary works of different nations when it comes to the dissemination of its image, and this country's people are unquestionably its primary source of image-related content.

The core of data warehouse technology is an information integration technology. Data warehouse is to obtain the original data from multiple information sources, and after sorting and processing, it is stored in the internal database of data warehouse. By providing access tools to users of data warehouse, it provides a unified, coordinated, and integrated information environment to support global decision-making process and comprehensive and in-depth management analysis [14].  Figure 2 shows the architecture of the data warehouse.

In the data warehouse, the source data comes from the existing production system, which is the operational data. The data sources that provide the source data can be various database management systems, data files in various formats, or external data sources. In the daily operation of the data warehouse, it is necessary to continuously monitor the status of the data warehouse, including the usage of system resources, the legality of user operations, data security, etc.

RETRACTED

In order to enable data warehouse users to effectively use the information in the data warehouse for complete and in-depth analysis and decision-making, the data warehouse system must provide users with a set of comprehensive data access and analysis tools. Data access and analysis tools should not only provide general data access functions, such as query, summary, and statistics, but also provide in-depth data analysis functions, namely, DM functions.

Pearson correlation coefficient measures the correlation degree of two variables by the ratio of covariance and standard deviation. Its value range is [1, 1]. The concrete method is to calculate the product of the difference between each variable and its mean value at each moment, and then add the product of the difference at each moment to get the mean value, as shown in formula (5):

(5) $$\begin{array}{c} \text{COV}\left(X,Y\right)=\frac{1}{n-1}\times \sum_{1}^{n}\left(X_{i}-\mu_{x}\right)\left(Y_{i}-\mu_{y}\right). \end{array}$$

If the result is positive, it means that the variables *X* and *Y* are positively correlated, and when it is 1, *X* and *Y* are completely consistent. If the result is negative, it means that *X* and *Y* are negatively correlated. 0 means that *X* has nothing to do with *Y*.

The main idea of NB (Naive Bayes) algorithm is to calculate the probability of the sample appearing in each category for each sample, and the category of the sample is the one with the highest probability. Bayesian theorem is to obtain the probability of event *A* under the condition of event *B* after the probability of event *B* is known, as shown in formula (6):

(6) $$\begin{array}{c} P\left(B|A\right)=\frac{P\left(A|B\right)\times P\left(B\right)}{P\left(A\right)}, \end{array}$$

where *P*(*B|A*) is the conditional probability of *A* occurring under the condition of *B*, and *P*(*A|B*) is the conditional probability of *B* occurring under the condition of *A*.

Evaluation index system is an organic whole composed of a number of interrelated and interacting evaluation indexes according to a certain hierarchical structure. Comprehensive evaluation is based on the index system to determine the evaluation object. The indicators must be representative and independent, the indicator system must be clear and concise, and each indicator must have a clear and relatively independent connotation, so as to better reflect the characteristics of a certain aspect of the evaluation object. Therefore, this topic first evaluates the existing evaluation indicators and checks the correlation of all system indicators, so as to reduce the indicators. As shown in Figure 3, it is a subject evaluation model.

RETRACTED

To determine the weight of each evaluation index, I first introduce the attribute reduction method of rough set, reduce these indexes, and create a system of indexes that is largely independent. The weight is known as the target weight because it is primarily based on data. The subjective and objective integral weights are obtained by combining the objective quantitative weight obtained by the approximate integration method with the evaluators' prior knowledge. The multi-layer fuzzy evaluation method is then combined to produce the comprehensive evaluation's final result after the weight has been established.

In a basin-shaped area on the fitness surface, the local search algorithm can find the basin floor representing the local extreme point when the time is enough. Let $\bar{\lambda }$ be the average local search time unit in one iteration of *H*, and one iteration of *G* be a time unit, then the time *T* spent for *n* iterations is:

(7) $$\begin{array}{c} T=\left(1+\bar{\lambda }\right)n. \end{array}$$

In some basins, the local search time *λ*_*i*_ from the starting point to the target area may exceed the allowable time *λ*, so that the target area cannot be reached in one iteration. Then the probability *P*_*λ*_ of*H* hitting the target area in one iteration is:

(8) $$\begin{array}{c} P_{\lambda }=P_{G}+\underset{i:\tau_{i}\neq 0,\lambda_{i}<\lambda }{\sum P_{i}}. \end{array}$$

Through the analysis of association rules, we can extract association rules that may not be detected between data, and then make corresponding decisions according to the obtained association rules. Increase the investment in one aspect, change the corresponding related factors, and avoid unnecessary waste of resources.

## 4. Experiment and Results

In this work, it is necessary to count the published status of articles, rather than the information of specific articles. First of all, the total number of scientific research papers published by each university every year is counted by using the three attributes of signature, unit name, and publication year in the published data.  Table 1 is an example of data after statistics and reduction of all articles published in some disciplines.  Figure 4 shows the trend of statistical results.

In addition to the general situation of teachers, the publication of high-level talents in various disciplines, including professors and associate professors, is also counted. Finally, because schools generally attach importance to the scientific research achievements of newly introduced talents, they will also count the number of papers published by newly introduced talents in various disciplines every year. It is worth noting that in the year when teachers started school, due to time, it was difficult to publish a sufficient number of articles, which could not reflect their true level. However, the articles published that year were probably based on the scientific research achievements made in the original unit.

RETRACTED

This section further discusses the influence of each attribute on the ranking relationship of students' total scores, and the relationship between students' scores in each course. As shown in Figure 5, it shows the changes of dietary consumption of the top and bottom students in one year.

It can be seen that the students with higher scores are roughly equal to those with lower scores. However, students with better grades are slightly better than those with lower grades in consumption frequency and consumption, especially in the first semester after enrollment. Students who can keep good habits in the first semester will be able to adapt to college life more quickly and get better grades more easily.

The validation of mixing effectiveness is shown in Table 2. NB algorithm is implemented in two situations: one is hybrid evolutionary algorithm and local search algorithm, and the other is nonhybrid evolutionary algorithm only. The extension method used in this section is single label extension.

From the experimental results, it can be seen that the result of running evolutionary algorithm combined with local search is better than that of running evolutionary algorithm alone. This also verifies the argument that the hybrid algorithm mentioned in the theory of hybrid evolutionary algorithm is superior to the general evolutionary algorithm.

In order to evaluate the performance of the NB algorithm, the substructure extension provided by Subdue is used in our experiment. As can be seen from Figure 6, when the substructure is expanded by adding one side, there may be multiple options. If the mutation is purely random, the algorithm will not converge for a long time, and the introduction of scaling algorithm can make the algorithm the focus.

In addition, the individual cooperation operator allows people to search for examples cooperatively; to some extent, it overcomes the phenomenon of example loss in the search process and significantly improves the understanding quality. With basically the same parameter settings, the experimental results of NB algorithm will not take too long, about 56.08 s, and the compression ratio is 0.897.

RETRACTED

Despite the fact that all of the indicators involved in this topic have a positive correlation, some of them actually have an inverse relationship. According to the so-called inverse relationship, the membership value decreases as the index value increases. For instance, if there are many teaching failures, we believe that the membership value will be higher the lower the number of teaching failures. Finally, as shown in Figure 7, the fuzzy membership value of each index of the prior evaluation object is determined.

This algorithm makes use of the index table structure, whose index key is the number of transactions in the transaction database. The index key, which is the length of the transaction, must be sorted before the index table is set. It is not possible to send many transactions to the memory at once; transactions must be sent to the memory in order of small to large. Because there are numerous transfers between the internal memory and the external memory during database scanning, it is necessary to scan the database from scratch before transferring each transaction to the internal memory. To locate the precise location of data that needs to be transferred to memory, a database is used. In addition, the index table's ability to quickly retrieve data from the database boosts the algorithm's effectiveness.

As we are looking at the selected data samples, each influencing factor is subdivided into different small quantitative values, which will lead to too much data and bring unnecessary problems to the analysis. We hope to get a single representative value. Therefore, here we introduce the weighted analysis commonly used in discipline evaluation. Combining the above treatment schemes, we get Figure 8.

In the process of gathering data, there are frequently omissions, vacancies, and other components. The results of mining will be heavily influenced and biased, leading to mining failure, if these projects are not managed. We clean these vacancies using data cleaning. The accomplishments of various disciplines can mainly be categorized into three groups: scientific research, teaching, and a heavyweight discipline that combines both scientific research and teaching. As the test attribute for the node, choose the attribute with the greatest information gain. As a result, classifying objects takes much less time overall.

There are distinct research areas for both comparative literature and world literature. The foundation of literature is multiethnic, multidisciplinary, and multicultural. To study the factual relationship or the aesthetic relationship without facts, two or more subjects are required. The study of comparative literature is based on an international perspective that transcends national, linguistic, cultural, and disciplinary boundaries. It examines the connections between literature from different nations and various literary phenomena as well as the general rules of literary development. The ultimate goal of world literature teaching and research, as well as the goal of literature comparison, is to aid us in understanding the fundamental rules of general literature and even human culture.

RETRACTED

## 5. Conclusion

Comparative literature differs from other literary studies in that it transcends time and space, which is reflected in the importance of its existence. Its research findings have greater universal validity and applicability in spiritual temperament because it transcends time and space. The spread of images is combined with the entire social system, which is interconnected and mutually restrained in terms of culture, politics, economy, etc. However, it is important to understand that image communication in the context of comparative literature is distinct from other types of image communication. Big data management and data analysis for schools have become widespread trends. In this course, the discipline construction of comparative literature and world literature is applied using DSS based on data warehouse. The concurrent completion and realization of the construction of the world literature discipline is based on DM technology, DSS comparative literature prototype system, and DM technology. The experimental results of the NB algorithm will not take too long, roughly 56.08 s, and the compression ratio is 0.897 with essentially the same parameter settings. For the purpose of providing a solid and trustworthy reference for our future investment decisions in scientific research and production, resource investment, and evaluation allocation, the application of DM technology in the field of subject evaluation has been preliminary completed.

## Figures and Tables

**Figure 1:** General framework of DSS for discipline construction of comparative literature and world literature.

**Figure 2:** Data warehouse architecture diagram.

**Figure 3:** Subject evaluation model.

**Figure 4:** Statistical result trend.

**Figure 5:** Average consumption is counted by month.

**Figure 6:** Comparison of experimental results.

**Figure 7:** Evaluation object fuzzy membership value.

**Figure 8:** Comprehensive data after data preprocessing.

**Table 1:** Examples of publication data of all academic papers.

Year	Discipline 1	Discipline 2	Discipline 3	Discipline 4	Discipline 5
2015	54	301	10	87	93
2016	53	351	8	81	96
2017	45	266	6	74	104
2018	41	286	9	56	109
2019	58	324	11	68	81
2020	44	365	4	61	100

RETRACTED

**Table 2:** Experimental results of mixed validation.

Data set	Mixed evolution	Individual evolution
1	0.261	0.288
2	0.863	0.896
3	0.902	0.908
4	0.823	0.833

## Data Availability

The data used to support the findings of this study can be obtained from the author upon request.

## References

[1] Baldwin C. (2014). Post-world war ii masculinities in British and American literature and culture: towards comparative masculinity studies. *Contemporary Women s Writing*.

[2] Mattana A. (2020). The allure of synthesis: science and the literary in comparative and world literature. *Comparative Critical Studies*.

[3] Schlumpf E. (2011). Intermediality, translation, comparative literature, and world literature. *CLCWeb - Comparative Literature and Culture*.

[4] Nie Tian. (2019). zhenzhao and the genesis of chinese ethical literary criticism. *Comparative Literature Studies*.

[5] Britto K. A (2012). Worlds within: national narratives and global connections in postcolonial writing. *Comparative Literature*.

[6] You L., Jiang H., Hu J. (2021). GPU-accelerated Faster Mean Shift with Euclidean distance metrics. https://arxiv.org/abs/2112.13891.

[7] Chen J., Ling F., Zhang Y., You T., Liu Y., Du X. (2022). Coverage path planning of heterogeneous unmanned aerial vehicles based on ant colony system. *Swarm and Evolutionary Computation*.

[8] Briceño X. (2016). Cosmopolitan desires: global modernity and world literature in latin america. *Comparative Literature*.

[9] Hoxby B. (2012). What was tragedy? the world we have lost, 1550–1795. *Comparative Literature*.

[10] Larsen S. E. (2019). Walter cohen, a history of european literature: the west and the world from antiquity to the present. *Comparative Critical Studies*.

[11] Zunshine L. (2020). Embodied social cognition and comparative literature. *Poetics Today*.

[12] Song B. (2018). On world literature, exile and cosmopolitanism: an interview with professor galin tihanov. *Foreign Literature Studies*.

[13] Shaytanov I. (2018). World literature as a challenge and ethical problem. *Foreign Literature Studies*.

[14] Wang L. (2018). Ethical literary criticism toward interdisciplinary studies and construction of world literature: a review of the 8th international symposium on ethical literary criticism. *Foreign Literature Studies*.

[15] Hassan A. R, Subasi A. (2017). A decision support system for automated identification of sleep stages from single-channel eeg signals. *Knowledge-Based Systems*.

[16] Kostuk K. J, Willoughby K. A. (2012). A decision support system for scheduling the canadian football league. *Interfaces*.

[17] Kheterpal S, Shanks A, Tremper K. K (2018). Impact of a novel multiparameter decision support system on intraoperative processes of care and postoperative outcomes. *Anesthesiology*.

RETRACTED

[18] Cartwright J, Caldwell C, Nebiker S, Knight R (2017). Putting flow–ecology relationships into practice: a decision-support system to assess fish community response to water-management scenarios. *Water*.

[19] Sim L. L. W., Ban K. H. K, Tan T. W, Sethi S. K, Loh T. P. (2017). Development of a clinical decision support system for diabetes care: a pilot study. *PLoS One*.

[20] Brown M., Black E., Asfaw D., Otu-Larbi F. (2017). Monitoring drought in Ghana using tamsat‐alert: a new decision support system. *Weather*.

